The article "The Pictorial Interview of Children's Metacognition and Executive Functions (PIC-ME): Cultural Adaptation for Ultra-Orthodox Jewish Populations" was published in 2023. Journal: Occup Ther Int.

# The Pictorial Interview of Children's Metacognition and Executive Functions (PIC-ME): Cultural Adaptation for Ultra-Orthodox Jewish Populations

**DOI:** 10.1155/2023/4832354

**Published:** 2023-04-14

**Authors:** Anat Golos, Jennifer R. Budman, Ayala Shterenshus, Ruthie Traub Bar-Ilan

**Affiliations:** ^1^Head of the Environment, Culture and Participation in the Community Research Laboratory, School of Occupational Therapy, Faculty of Medicine of the Hebrew University, Jerusalem, Israel; ^2^School of Occupational Therapy, Faculty of Medicine of the Hebrew University, Jerusalem, Israel; ^3^School of Occupational Therapy, Cognitive-Functional Rehabilitation in Context Laboratory, Faculty of Medicine of the Hebrew University, Jerusalem, Israel

## Abstract

**Introduction:**

Executive functions (EFs) are strongly linked to attention deficit hyperactivity disorder (ADHD). The pictorial interview of children's metacognition and executive functions (PIC-ME) assesses children's self-perceptions regarding their EF. This study is aimed at describing the cultural adaptation of the PIC-ME to the ultra-Orthodox (UO) Jewish population in Israel.

**Method:**

In the first of three stages, 30 occupational therapists, who were experienced in working with children with ADHD from the UO population, completed a questionnaire about the suitability of PIC-ME for the UO community. In the second stage, six therapists participated in a focus group to discuss the recommendations and the adaptations made following the first stage. In the third stage, 20 UO children aged 5–10 participated in the tool validation process.

**Results:**

First stage: most of the items of the original tool were found to be appropriate in representing the EFs of UO children and did not need to be adapted. No significant differences were found between the boys' and girls' versions regarding the tool's adaptability. However, most of the therapists suggested that the pictures in both versions needed adaptations. Second stage: additional recommendations led to the development of a final adapted version. Third stage: over 70 percent agreement was found among UO children regarding the clarity of the adapted pictures. No significant differences were found between boys and girls or between age groups.

**Conclusions:**

This study presented wide agreement on the necessity for cultural adaptation of the PIC-ME to the UO population and described the adaptation process. Based on its face validity, the UO version may be a useful tool to assess the self-perception of EF among UO children. Further studies are needed to assess its psychometric properties and its usefulness as an outcome measure. The study findings may contribute to the cultural adaptation of other tools for culturally distinct populations.

## 1. Introduction

Executive functions (EFs) are defined as a set of interrelated higher-level neurocognitive, self-regulatory processes, involving cognition, emotions, and behaviors [1–3]. EFs are responsible for directing and coordinating one's actions toward future self-serving goals [4]. Subcomponents of EFs frequently mentioned in the literature are inhibition, initiation, mental flexibility/shifting, working memory, planning, organization, and self-monitoring [1, 5]. Deficits in EFs (EFDs) are present in almost every health condition that affects information processing, learning, and brain functions, even in the absence of frontal lobe injury [6]. One of the health conditions that is strongly linked to EFD is attention-deficit hyperactivity disorder (ADHD) [7].

ADHD is a lifelong neurodevelopmental disorder (NDD), characterized by core symptoms of inattention, hyperactivity, and impulsivity [8]. It is associated with many functional impairments in everyday activities, challenges in social interactions, and academic underachievement [9]. The prevalence of ADHD has been estimated at around 5.3% to 7.2% among school-aged children [10, 11]. Studies consistently associate ADHD with adverse life outcomes in multiple functional domains [12, 13], as well as decreased quality of life (QoL) [14–16]. ADHD is thus conceptualized as a chronic neuropsychiatric health condition that requires lifelong management [17, 18]. Self-awareness (SA) of personal strengths, challenges, and strategies is central to adaptive self-management of chronic health conditions such as ADHD [19, 20]. The growing body of evidence demonstrating the significant impact of EFD on participation and QoL among people with ADHD provides the rationale for developing assessments along with evidence-based interventions which target EFD in the context of participation.

One of the most up-to-date interventions for ADHD is the cognitive–functional intervention (Cog-Fun) [21]. It targets the SA of EFD in occupational contexts, incorporating neurocognitive rehabilitation principles within an occupational therapy intervention framework. Cog-Fun employs four central change components: metacognitive learning and executive strategies acquisition, occupation centeredness, environmental support, and positive engagement [20]. Several studies of children with ADHD using the Cog-Fun intervention indicated a positive effect on executive functioning and quality of life, as well as a reduction of ADHD symptoms and EFDs, as reported by parents. In a randomized controlled trial, these results were maintained after a three-month follow-up [22, 23]. In a recent systematic review on the effectiveness of pediatric occupational interventions, the Cog-Fun was rated as a high-quality evidence base, and it was recommended for use among children with ADHD [24]. As mentioned, one of the key principles of the Cog-Fun is metacognitive learning integrated with executive strategies acquisition, in the context of playful activities. The ability to identify strengths and challenges in EFs can be a powerful agent in personal goal setting and in transferring strategies to daily life [25]. Therefore, for children with ADHD, a collaborative child- and family-centered inquiry into the child's EF profile may improve ADHD interventions [26].

Assessments of children's EFDs are usually based on parents' and/or teachers' reports using questionnaires [27]. They, however, see the child from their own perspective and usually in a specific context, which may lead to bias [28]; as a result, there are often discrepancies between reporters [29]. Moreover, in many evaluation processes, the children's own perspective concerning their health condition is absent. Interventions emphasizing integration from a client-centered perspective should seek to understand children's perspectives regarding their health condition, challenges, strengths, and resources.

Several child self-rating tools on cognitive functioning have been developed [30], yet the literature has been inconclusive regarding young children's ability to identify challenges and set goals. Moreover, studies among children with ADHD demonstrate strong evidence for the overestimation of competence known as positive illusory bias (PIB) regarding academic, social [31], and cognitive domains [32]. However, children with ADHD were able to rate their occupational competence in everyday activities using a pictorial assessment [33]. Children were also able to use their self-perception of challenges and abilities for goal setting [34].

A barrier in the process of promoting the child's SA in the Cog-Fun approach was the absence of a child self-report assessment regarding EFDs and strengths. Therefore, the pictorial interview of children's metacognition and executive functions (PIC–ME) [35] was developed to evaluate the self-perception of EFDs and strengths among young children with ADHD (aged 5–10 years) in a variety of occupational contexts. In addition, parents also completed the PIC-ME questionnaire regarding their child's EFDs and strengths in daily life. The PIC-ME item development was based on Brown's comprehensive clinical model [1], including six EF clusters that characterize the challenges facing people with ADHD in real-world contexts. The PIC-ME development process and its psychometric properties were described in the Traub Bar-Ilan et al. study (2018) [26], which supported the reliability and validity of the PIC-ME as a child-centered assessment of EF challenges and strengths for children with and without ADHD. The study results demonstrated high internal consistency for the total PIC-ME EFD score, with a high and significant correlation between the PIC-ME parent total score and the Global Executive Composite of the Behavior Rating Inventory of Executive Function (BRIEF) [5], thus supporting the concurrent validity of the PIC-ME assessment. Moreover, significant differences in all scales and total EF scores of the parental PIC-ME EFD ratings showed that parents of children with ADHD identified significantly higher percentages of EF challenges, compared to parents of typically developing children. These findings supported the PIC–ME's construct validity in identifying EF challenges among known groups with EFDs (for more details, see the Measures section).

Nevertheless, some concerns were raised regarding the reliability of the PIC-ME scales, with less consistent results in children's self-ratings. One factor was a strong PIB tendency among the children with ADHD, in congruence to the literature showing that self-ratings of children with ADHD significantly differ from those of their parents or teachers, who identify more challenges than their children [31, 32, 36, 37]. Another factor that may explain at least some of the discrepancies found in the children's self-report, which was not mentioned by the authors, is the different ethnocultural backgrounds of the families who participated in the study. The PIC-ME pictures were designed for the general population; hence, the study sample was comprised of children from varied ethnocultural backgrounds, including religious and ultra-Orthodox (UO) Jewish families. However, the items were not specifically adapted for these populations.

The UO Jewish population is a minority group of highly religious individuals who belong to an internally cohesive and externally insulated community with a commitment to halacha, a body of rabbinic Jewish laws and customs [38]. They display characteristics similar to other highly religious populations [39], in that their values, beliefs, and behaviors are greatly influenced by their community's cultural codes and obligations [40, 41], which influence all aspects of daily living [41, 42]. UO members are characterized by cultural conservatism, along with fixed boundaries between themselves and the general population to minimize outside influences [43]. They usually live in segregated communities and tend to have larger-than-average families and lower-than-average incomes [44]. Previous studies found in the literature have emphasized the need for cultural adaptation for the UO population in order to achieve meaningful results and build an effective therapeutic relationship between the occupational therapist and UO clients. For example, Golos et al. [42] emphasized the need for cultural adaptation in occupational therapy, which included understanding the effects of beliefs regarding health and education, developing culturally sensitive assessments and interventions for UO children, making adaptations in the assessment or intervention process, and setting goals that are meaningful and relevant to clients and their families. To address the needs of populations with unique cultural characteristics, such as the UO community, assessment instruments must be tailored and sensitive to different cultural or ethnic populations [45, 46]. Based on the use of the PIC-ME in Israel as part of the Cog-Fun intervention for children with ADHD, therapists have voiced a need to adapt the graphic content and contexts of the PIC-ME child report accordingly.

The cultural fit of an evaluation tool is defined as the extent to which the items in the translated or adapted tool are representative of the tool's original items [47]. Cultural equivalence in addressing an assessment tool includes three components: content (concepts, items, and semantics), administration (operational procedures), and measurements such as validity [48]. Additionally, an adaptation of assessment tools requires an understanding of the content world of the specific target population. In line with this argument, it was found that when targeting the participation of UO children, there is a need to understand their specific cultural values and beliefs [49]. The measurement component of the cultural adaptation process includes validity assessment. An initial measure of validity is face validity, defined as the degree to which the tool's items adequately reflect the assessment objectives and the structure being measured [47] when evaluated by a potential target group [50].

Based on a review of the literature and the needs of the specific population, this study is aimed at culturally adapting the PIC-ME to UO children aged 5–10, who often participate in occupational therapy intervention. The specific research objectives were to examine the following: (a) therapists' attitudes toward the suitability of the PIC-ME for UO children and their views concerning the need for its cultural adaptation and for the kind of adaptation required; (b) therapists' attitudes regarding the adapted version of the tool; and (c) the tool's face validity as tested among 20 UO children with typical development.

## 2. Materials and Methods

### 2.1. Study Design

A mixed-method one-group study design was employed, using both quantitative descriptive methods and qualitative content analysis of data. Mixed-method research is the process of integrating quantitative and qualitative data collection and analysis to generate metainferences beyond what either approach could do alone [51]. This research design holds the promise of richer and more comprehensive research solutions. Its rigor in this study was noted in three dimensions: rationale and description (e.g., description of data collection and analysis); a transparent and detailed description of method and results; and integration of quantitative and qualitative components [52]. This study consisted of three stages. The first stage included collecting descriptive information through a questionnaire for occupational therapists. The second stage included a focus group with therapists, and the third stage included collecting descriptive information from UO children.

### 2.2. Participants

In the first stage of this study, a questionnaire was completed by 30 occupational therapists, all of whom were certified in the Cog-Fun approach and had experience in treating children with ADHD and UO children. They all expressed consent to participate in this study. They were all women, with professional experience as occupational therapists (range of 4-30 years, *M* = 9.95, SD = 5.87). Most of them (63.3%, *n* = 19) held a bachelor's degree, and the others (33.6%, *n* = 11) had a master's degree. Most of them (83.3%, *n* = 25) were born in Israel and spoke Hebrew; the others spoke English. All of them defined themselves as Jewish; most of them were UO (*n* = 18, 60%), with others identifying as religious or secular (*n* = 8, 26.7%; *n* = 4, 13.3%. Occupational therapists from stage one were asked if they were interested in participating in stage two. In the second stage of the study, six therapists who displayed interest from stage one agreed to participate and were then included in a focus group. In the third stage, 20 UO children aged 5–10 (10 boys and 10 girls) participated, with two children from each gender (boy and girl) serving as samples in each age group (5-6, 7-8, 8-9, and 9-10 years). The inclusion criteria were children with typical development attending regular educational settings. The exclusion criterion was diagnosis of a specific health condition (brain injury, cerebral palsy, Tourette's syndrome, epilepsy, ASD, ADHD, psychiatric disorder, or severe sensory impairments such as deafness and blindness) according to parents' reports.

### 2.3. Procedure

Approval for this study was obtained from the Ethics Committee of the Hebrew University (No. 08052019). In the first stage of the study, an email was sent to a list of occupational therapists certified in using the Cog-Fun intervention for children with ADHD. Participants who expressed interest contacted one of the study's researchers for additional explanation. Following written consent to participate in the study, they completed the questionnaire. The information that was collected from the questionnaires was analyzed and discussed by the research team, which included two UO occupational therapists experienced in working with children with ADHD, one of the tool's developers, and a lead researcher on behalf of the academic institution. Based on the data, a few statements were changed, and adaptations were recommended in most of the pictures. The tool was then sent to the original graphic designer for modifications. Following those changes, the first adapted version of the PIC-ME was formulated.

In the second stage, a focus group was convened with consenting therapists from stage one who agreed to participate in this stage, and the first adapted version was presented. The participants were asked to express their opinions on the appropriateness of this version for the UO population, as well as to suggest additional adaptations. The meeting was recorded and transcribed. The content was then discussed by the research team, and key themes were identified. Following this phase, further adaptations were carried out, and a final version was formulated for use in the third stage of the study.

In the third stage, the request for the participation of typically developed UO children was advertised on bulletin boards in nearby UO educational settings. Participants were recruited through a convenience sample. Having considered the study's exclusion and inclusion criteria, parents were asked for their child's age and gender. The study was explained, and parents gave their written and oral consent. Oral consent was also obtained from the children, and they were asked questions to measure their understanding of the PIC-ME-adapted items presented to them, using a questionnaire that was developed for the purpose of this study.

### 2.4. Measures

#### 2.4.1. Pictorial Interview of Children's Metacognition and Executive Functions (PIC-ME)

The PIC-ME [35] was designed to evaluate the self-perception of EFDs and strengths among young children (aged 5–10 years) with ADHD in occupational contexts. It consists of 44 items, each described by a general sentence (pictorial script), and accompanied by pictures and statements describing daily activities and situations. Of these, 34 items representing EF challenges are grouped into six scales delineated from Brown's model [1]: activation (prioritizing tasks and getting started on tasks); focus (concentrating on a stimulus, maintaining focus on a given task, ignoring distractions, and shifting focus to new tasks); effort (regulating alertness and speed, sustaining effort); emotion (managing frustration and modulating emotions); memory (using working memory and accessing recall); and action (inhibitory control and self-monitoring). Ten more items represent EF strengths. Administration of the tool includes several stages, depending on the child's responses. The child is asked whether the situation depicted in each item (pictorial script) happens to him or her as well (1 = “yes,” 0 = “no”). A positive answer is followed by more in-depth questioning regarding frequency (sometimes and often), context (home, school, or community), whether it bothers the child, and whether the child wants to change it. The number of “yes” answers is summed up for all EF challenges and for each EF scale, divided by the number of items on the scale, and multiplied by 100 to obtain a score ranging from 0 to 100. A goal scale is calculated by summing up the number of EF items that the child wants to change, ranging from 0 to 34. The PIC-ME includes boys' and girls' versions, as well as a separate corresponding parental version of the PIC-ME questionnaire.

A study sample of 100 children diagnosed with ADHD (64 boys and 36 girls) and 44 typically developing children (22 boys and 22 girls) participated, in order to establish the reliability and validity of the PIC-ME [26]. The results supported the psychometric properties of the PIC-ME, with high internal consistency for both child and parent ratings for the total EFD PIC-ME score (*α* = .953 and .914, respectively). Additionally, a high correlation with the Behavior Rating Inventory of Executive Function (BRIEF; *r* = .72) was found, as well as significant differences between parents of children with and without ADHD on all PIC–ME EFD scales of the parent PIC-ME version (*p* < .0001). No differences were found between groups on the parent version regarding the strength scale. However, children with ADHD rated their strengths significantly lower than typically developing children [26].

#### 2.4.2. Questionnaire for Therapists on the Suitability of PIC-ME for UO Populations

As part of this study, a questionnaire was developed to examine therapists' views on the suitability of the tool for UO children aged 5–10. It consisted of 15 questions related to demographics and professional information, along with open-ended questions. For example, age, religiosity level, professional education, using the Cog-Fun protocol intervention, and service recipients' characteristics. The suitability of the items' content and pictures for UO children was rated using a scale of 1–5 (1 = “not at all,” 2 = “slightly,” 3 = “partially,” 4 = “largely,” and 5=“absolutely” suitable). Specifically, the therapists were required to rate the item's representation of the functioning of UO children aged 5-10, and how clear the statements and pictures are to these children. Item examples were as follows: “He/She can't find his stuff,” “He/She has a hard time waiting for his turn” and “He/She chats a lot during lessons.”

#### 2.4.3. Questionnaire for UO Children on the Clarity of PIC-ME Items

This questionnaire was developed for this study to assess the validity of the adapted version of the tool among UO children aged 5–10 years with typical development. It consisted of four questions presented to the child while viewing the pictures and statements. For each picture, the child was asked the following: (1) “What do you think the child in the picture is doing?” And the child's response was recorded; (2) “One of the children told me that...” (the researcher read aloud the statement, for example, “He interrupts Mom as she talks on the phone”); “Do you think the picture illustrates what I just read?” And the child's answer was marked (“yes/maybe/no”); (3) “Does the child in the picture resemble one of the children you know?” And the child's answer was marked (“yes/maybe/ no”); and (4) If the child answered “no,” the researcher asked him: “How is it different?”; and the child's response was recorded, as well as any additional comments.

### 2.5. Statistical Analysis

The quantitative data were analyzed using the Statistical Package for the Social Sciences (SPSS v. 25; IBM). The significance level was set at 0.05. Descriptive analysis was used to describe the sample characteristics, means, standard deviation, frequencies, and percentages. In order to calculate a general mean score of the items in the therapist questionnaire, dichotomous variables were defined (1 = “largely” and “absolutely”; 0 = “not at all,” “slightly,” and “partially”). In the children's questionnaire, the variables were defined as (0 = “maybe” and “no”; 1 = “yes”). The Mann–Whitney nonparametric test was used to examine differences between boys and girls. Qualitative information was analyzed using content analysis, identifying key themes according to Krueger and Casey [53]. The process included triangulation of the data as recommended by Tracy [54]; four of the researchers, two of whom identified as UO members, converged on the same conclusions, thus improving the credibility of the current study.

## 3. Results

### 3.1. Stage I

All participants agreed that the PIC-ME tool was “moderately important” to “very important” for raising awareness of EFDs and for identifying functional goals during the intervention, including UO children with ADHD. Also, they stated that all PIC-ME items accurately represented the EFDs and strengths of children with ADHD. However, they reported that the original tool was a barrier, since it did not enable UO children to identify with the various characters and occupations presented. Overall, more than half of the participants (*n* = 17, 56.17%) avoided using the tool among the UO population due to its cultural incompatibility. The participants indicated a high consensus (over 70%) regarding the extent to which the items (“to a large extent” and “absolutely”) represented the EFs of UO children aged 5–10, meaning that the representation of the EFs' items to this population was also applicable. However, a similar consensus (over 70%) indicated that the depictions of the items should be adapted to the UO population; most of the pictures in the tool were judged less than suitable (“partially,” “slightly,” or “not at all”). The Mann–Whitney test showed no significant differences between the boys' and girls' versions regarding the degree to which the items represented UO children (boys: *M* = 0.87, SD = 0.22; girls: *M* = 0.88, SD = 0.16; *Z* = 0.26, *p* > 0.05), as well as regarding the low suitability of the pictures (boys: *M* = 0.37, SD = 0.32; girls: *M* = 0.25, SD = 0.25; *Z* = 0.47, *p* > 0.05). According to these results, it seemed that both versions required similar pictorial adaptations.

segregation in educational, play, and leisure activities; a dress code familiar to UO culture (e.g., long skirts and shirts for girls; yarmulkas for boys); renaming the girl with a more common name in the UO population; and depiction of activities more common among UO boys or girls (e.g., playing a football game, for the boys' version; going to the school secretariat and forgetting that the teacher asked to bring pages to class for the girls' version). In addition, it was recommended to omit activities not appropriate for the UO population (e.g., playing on a PlayStation and watching TV), to add statements that include familiar cultural activities, and to change the depicted background environment (e.g., omitting TV in the home). Using this information, several statements and pictures were modified, and a first adapted version was formulated.

### 3.2. Stage II

Participants in the focus group were presented with the first adapted version of the tool and were asked to give feedback and suggest additional changes. All the participants in the focus group supported the initial changes made, recommended additional changes, and expressed a desire for the final adapted version to be used among UO children. The qualitative information that was collected during the two stages of the study was analyzed by the research team and divided into three themes: characteristics of the depicted character, their environments, and their occupations. This information is summarized in Table 1; examples of adapted pictures and statements are presented in Figures 1–4. Following this stage, further adaptations were carried out, and a final version was formulated for use in the third stage of the study.

#### 3.2.1. Characteristics

The changes made in the characters depicted in the tool were reported as indeed appropriate to the UO population. Additionally, the participants suggested changing the appearance of the depicted educational staff, as well as the clothing style of three of the characters.

#### 3.2.2. Environments

Participants discussed the physical environments depicted inside and outside the home. They supported the changes made to the tool in portraying the home environment and suggested adding other objects. The participants also agreed with the changes made to the environment outside the home and suggested further changes.

#### 3.2.3. Occupations

Participants noted the importance of depicting occupations visibly relating to customs and religious ceremonies characteristic of UO culture. Due to the diverse nature of the UO population, it was recommended to make changes only to items which represent a “banned” or unacceptable activity in this population (such as watching TV or engaging in activities with no gender separation) and to leave neutral depictions which do not contradict common UO values and norms. Participants agreed that specific religious statements should be added, and recommended further changes to play, leisure, and learning activities. Based on these results, a final adapted version was developed.

### 3.3. Stage III

The initial validity of the final version of the adapted tool was evaluated by presenting it to 20 UO children aged 5–10 years with typical development. The results indicated that most of the children (over 75%) agreed that the general statements described what they saw in the pictures. The percentage of positive responses (answering “yes” to the following question: “Does the picture illustrate what I just read?”) to all questions was 89%. These findings may indicate that the children understood the depiction of each of the items. Additionally, most of the children (over 70%) indicated that what happened in the pictures could happen to one of the children they know in relation to most of the items (39 out of 44). The percentage of their positive responses (answering “yes” to the following question: “Does the child in the picture resemble one of the children you know?”) to all the questions was 84%. These findings may indicate that the items represent activities familiar to children, so they readily understand them.

The results of examining differences between children from different age groups in understanding the pictures indicated that children aged 8–10 years were more likely to respond positively than children aged 5–7 years (97% and 78%, respectively). In addition, younger children described what they saw in the pictures as a story and even added details, without referring to the written statement and its meaning; this was in contrast to older children, who referred to the written statement along with describing what they saw in the picture. The Mann–Whitney test results indicated no significant differences between boys and girls in picture comprehension (boys: *M* = 0.87, SD = 0.15; girls: *M* = 0.91, SD = 0.08; *Z* = 0.53, *p* > 0.05). Additionally, no differences were found between boys and girls regarding their belief that what was depicted in the picture can happen to a boy or girl they know (boys: *M* = 0.82, SD = 0.18; girls: *M* = 0.86, SD = 0.15; *Z* = 0.34, *p* > 0.05). In conclusion, both boys and girls understood what was shown in the items and reported that the items were familiar to them.

## 4. Discussion

The aim of this study was to investigate the suitability of the PIC-ME for the UO population and to determine which cultural adaptations are needed in the PIC-ME assessment for children aged 5–10 years in the UO population. The UO population is a minority group of highly religious individuals with characteristics similar to other highly religious populations [39]. They are characterized by cultural conservatism in an insulated and segregated community, and they subscribe to a specific set of sacred principles and writings which are all encompassing [38, 40–43]. The UO population has been studied in the literature as representatives of highly religious populations in general [40], and this group may therefore provide information relevant to other highly religious populations in relation to the cultural adaptation of psychometrics.

The study included three stages. In the first stage, the majority of occupational therapists participating in the study agreed that there was a need for cultural adaptation of the PIC-ME for the UO population, and they offered suggestions to that end. Accordingly, a first adapted version was developed, which was used in stage II, where a focus group of occupational therapists met to assess the adapted version. Qualitative content analysis was performed, and a final adapted version was developed and used in stage III, which examined the face validity of the tool among typically developing children from the UO population.

Half of the participating therapists in stage I reported that they refrained from using the original PIC-ME tool among their UO clients, due to its cultural unsuitability for this population. Thus, it became apparent that the tool needed to be culturally adapted for this population in order to allow for more inclusive evaluation and intervention. This need was also supported by Hammell [55], who emphasizes the importance of acknowledging cultural differences, in order to promote inclusiveness and client-centered health care among diverse populations and improve intervention outcomes. Cultural adaptation of psychometrics to specific populations is critical for capturing the client's subjective experience. Culture may affect perceptions and understanding of concepts, and cultural miscommunication can elicit responses that misrepresent the true nature of the client's experience. In addition, valid and reliable measurements are needed for research-based intervention, indicating a need to measure the psychometric properties of culturally adapted measurements [56]. An example of examining psychometric properties of culturally adapted tool was described by Vall et al., [57], relating to the Dominic4 questionnaire, a pictorial structured tool for assessing mental disorder among children, which was also culturally adapted to African-American children, called the Terry questionnaire. This need was reflected as well in the occupational therapists' high regard for the PICME tool while at the same time refraining from using it because of cultural unsuitability.

More specifically, our findings indicated a high consensus among participating therapists (>70%) that there was no need to adapt the tool's items for this population regarding EFs' representation and strengths. A possible explanation for this may be that the actual items featured in the tool (e.g., difficulty in planning and organizing) [58] are representative of common EF challenges among children with ADHD, including the UO population [59]. Specifically, the items' phrasings were seen by participants as “general statements” of EF challenges relevant to children from a variety of sectors, including the UO population. Therefore, although the tool has not been validated among children from the UO population, the phrasing of the items may be considered suitable for children in the UO population. This was in line with Gjersing et al. [60], who argued that it is important to first establish the applicability of the concepts being measured to the target population, before implementing cultural adaptations to the measuring tool.

Subsequently, regarding the tool's pictures, more than half of the therapists reported the need for their cultural adaptation. Content analysis of the descriptive and qualitative data indicated three key themes for adaptation: the characters, environments, and occupations. Regarding the characters, the need for gender segregation was suggested in educational settings, play, and leisure activities. Characters' clothing adaptation includes adding a yarmulka on the head of males, hair covering for adult women, and modest attire according to the UO dress codes. These recommendations are consistent with the literature describing cultural sensitivities and norms regarding dress codes and gender segregation [39, 61], which are characteristic of the UO population [62, 63]. These dress-code adaptations have also been integrated into other evaluation tools for similar reasons, such as the Katenberger diagnosis tool [64]. Regarding the environment, pictures representing leisure activities with a television and/or computer were deemed culturally unsuitable for the UO population. These suggestions are in line with the literature reporting that television and computer use is less common in most UO homes [65]. Our participants suggested replacing these pictures with a library or street as a more familiar leisure environment among the UO population. Regarding the activities, pictures of people watching television and using the computer were suggested for the omission, for the reasons stated above [65]; suggested replacements were pictures representing behavioral activities during typical religious customs and rituals, such as the traditional response delay during Kiddush, reciting blessings over food before eating, and waiting until after washing hands before eating bread. These suggestions are in line with the findings of Golos and Weintraub [66], where educational staff noted some of those activities as part of the children's participation in the UO educational setting in particular and an integral part of life participation of these children in general. Additionally, dress codes, gender roles, environments, and activities commonly reflect cultural sensitivities among various highly religious populations, similar to the UO population [39]. Thus, it may be important to consider cultural adaptations of psychometrics and interventions among such groups.

The study findings indicated nonsignificant differences between the boys' and girls' versions of the tool, in relation to the degree of representation of the items, the clarity of the pictures, and the statements describing them. These findings suggest that the adjustments of the pictures and statements in both versions were similar. However, qualitative data expressed the need for specific adjustments regarding gender. For example, it was suggested to change the girl's name to a more common name in this population. It was also proposed to show gender-specific activities according to the norms of the culture. For example, it was suggested to add activities such as reading a book, playing a football game, and building a camp and campfire to the boys' version. In contrast, it was suggested to omit homework as an activity in the boys' version, because they typically complete their educational assignments at their school, which ends later than the girls' school. These findings are in line with research that examined the impact of culture and gender on kindergarten children's participation and found that cultural values may influence gender expectations as well as children's participation in daily activities [49]. Since our study is the first to examine gender differences in relation to the PIC-ME items, there is a need to further examine these differences across a variety of populations.

The process of the tool's cultural adaptation in this study included aspects related to the content of the pictures and the characters' dress code. An adapted version for the UO target population was created and used in stage III, to test face validity among typically developing children from the UO population. Content adjustment and initial psychometric testing of the adapted tool were based on recommendations in the literature regarding the cultural adaptation process required for assessment tools [48], and the same principles may also be applied to the adaptation of other tools to a variety of populations. This included measuring the face validity of the adapted PIC-ME for UO children, by examining the degree to which the participants understood the tool's statements and depictions after the cultural adaptations were made. Similar confirmation was performed in research by Paulisso et al. [67]. Results indicated that most participants agreed that the statements described what they saw in the pictures. In addition, the participants expressed that what they saw in the picture is common and can happen to someone they know, which may indicate that the pictures represent activities familiar to them. Kayihan et al. [68] described the cultural adaptation process of a sensory profile assessment for Turkish children with autism using parents' responses. They concluded that the cultural adaptation process needs to reflect the characteristics and needs of various cultural groups by using activities that are familiar to the clients. An additional example of cultural adaptation of an assessment is the perceived efficacy and goal setting (PEGS) tool assessing a child's ability to participate in daily activities, which was adapted to a German-speaking region in Australia. This study included 42 children aged 5-10, with their parents and teachers, who added specific culturally relevant activities in order to adapt the content to the children's daily lives within their cultural context [69]. As face validity measures whether the items of each domain are sensible, appropriate, and relevant to the people who use the measure on a day-to-day basis, these findings may support the initial internal validity of the tool and help support the assumption that the items reflect what is being measured by the tool [47, 70]. In this study, the face validity was measured based on an assessment by a potential group of subjects [50] typically developing UO children at the age for which the tool is intended. However, since the tool is intended for children with EFDs, further validity studies are required among this group. Our process of examining face validity in this study was similar to that of Lopes [71], who evaluated the self-assessment tool, the pictorial scale for perceived movement skill competence for young children (PMSC), among Portuguese children to assess its cultural relevance. The children were asked about the degree to which they understood what was happening in the pictures (e.g., “What skill/activity is shown in the picture?”). The findings of our study indicated that most children understood what was shown in the pictures [72], which supported the assumption that their content adaptation was successful.

Regarding different age groups, a majority of children in all age groups understood the statements and content in the pictures. Positive responses increased with the child's age, explained by the fact that older children are generally exposed to a greater variety of situations and behaviors in daily life, and their level of awareness of their own behavior is higher compared to younger children [73]. Differences in understanding specific questions between children from different age groups were also noted in another study that examined the psychometric properties of other pictorial instruments [57]. Answers regarding what they saw happening in the pictures were thus reflected by the developmental age of the children. Children in the younger age groups referred to concrete details in the pictures and, sometimes, also added their own details, without reference to the meaning of the descriptive statement. This was typical of younger children, who tend to focus on concrete details and have difficulty understanding more abstract ideas [72]. The fact that younger children did not use the general statements describing the pictures, or relate to text contained within the images, can also be explained by that age group, having not yet acquired reading skills [74].

Results indicated that there were no significant differences between genders in understanding the content in the pictures; therefore, the same cultural adaptations could be made to the boys' and girls' versions. However, further studies on validity regarding gender and ages are required.

### 4.1. Clinical Implications

Most participants in the two first stages of the study reported avoiding the use of the PIC-ME with their clients in the UO population or reported making adaptations that were not evidence based. This indicates that adapting the tool for clinical use among the UO population will support culturally competent occupational therapy practice, thus improving the quality of services and health outcomes among minority populations [59]. In addition, as there is a diversity of cultural sensitivities within subgroups of the UO population, it was decided that the adaptations should include only issues relating to traditional prohibitions common to all subgroups, such as modesty and gender segregation [61].

The present study focused on the cultural adaptation of a specific assessment tool to a specific population. However, characteristics of the UO population have been used to represent other highly religious groups and may therefore provide insight regarding cultural adaptations for those groups as well. This stresses the importance of valid and reliable adaptation of assessment tools and other protocols for minority groups and cultures, to ensure a culturally sensitive and evidence-based clinical practice. Our results helped create a culturally adapted version of an assessment tool that may be used clinically for assessment and intervention among UO children. The adaptation may also serve as a basis for further research.

### 4.2. Research Limitations and Recommendations for Further Research

Some limitations of this study may be noted. Firstly, in stage III, UO children were freely asked by the researchers what they saw in the pictures, without the written statements being read to them. This fact may have influenced the responses made by the younger children who were not able to read the statements, in contrast to the older children who could read the statements presented with the pictures. Secondly, participants included 20 typically developing children, one male and one female from each age group, through a convenience sampling from an urban setting. This may not be fully representative of children from the UO population, and further studies are recommended with a larger sample of this population. As face validity is an initial measure of validity, further comparative studies are recommended, such as measuring the validity of the tool among children with and without ADHD, from the UO population and from the general population, and examining if there may be differences among genders or ages of children from the UO population. In addition, the current research focused on the cultural adaptation of the PIC-ME child report only, according to the recommendations of the occupational therapists. Further research is recommended to assess the need for cultural adaptation of the PIC-ME parent report.

## 5. Conclusions

This study included a cultural adaptation of the PIC-ME tool for children from the UO population, based on clinical necessity. The data was collected through reporting and opinions of experienced occupational therapists, as well as through an examination of face validity among children from the target population. In adapting the tool, the content of the items was changed by adapting them to fit the values, norms, and lifestyle of the target population. The adjustment may enable the tool to be used for the assessment and intervention of target populations and specifically assess the self-perception of UO children aged 5–10 concerning the strengths and challenges of their EFs. Further studies are needed to establish the psychometric properties of the adapted tool and to examine its effectiveness as an intervention tool for this population. Cultural adaptations made in this study can also be applied to the adaptation of assessment tools or even intervention protocols among this population, as well as adaptation to other religious or traditional populations. The application of this process may serve as an example for similar adaptation of various tools required for assessing a range of functions among other populations with unique cultural characteristics.

## Figures and Tables

**Figure 1:** “Daniel does not finish eating his sandwich during the meal break.”

**Figure 2:** “Dina forgets her food.”

**Figure 3:** “Dina finds it hard to remain silent during the Shabbat Kiddush.”

**Figure 4:** “Daniel lies and dreams despite being repeatedly told to learn Torah.”

**Table 1:** Summary of themes, explanations, and examples as reported by participants in stages I and II of the study.

Theme	Explanation	Changes and adaptations (examples)
Characters	Adaptation of the characters (name, appearance, and clothing style)	(i) Renaming the girl (from Daniel to Dina) (ii) Changing the appearance of educational staff (iii) Adding modest clothing for girls and women (long skirts and shirts and adding a headdress for women) (iv) Adding a beard for men and yarmulkas for boys and men

Environments	Adapting home environment (use of suitable objects)	(i) Omitting TV and computer (ii) Adding a library
	Adapting outside environment	(i) Changing the playing environment (ii) Changing the leisure environment from a mall to a street (iii) Replacement of a zoo with an amusement park

Occupations (activities)	Adding occupations related to typical religious customs and rituals	(i) Omitting unacceptable activities (playing on PlayStation, watching TV, and using a computer) and replacing them with activities such as reading a book or a newspaper (ii) Presenting separate activities for boys and girls (e.g., adding activities such as football game, building a camp and campfire; omitting activity of complete homework for the boys' version; bringing photocopied pages to class for the girls' version) (iii) A statement was added regarding the need to delay a response during Kiddush (a blessing recited over wine or grape juice to sanctify the Shabbat and Jewish holidays), by remaining silent and waiting in line for the ritual washing of hands before eating bread (iv) Adding a statement that addresses the need for persistence while studying (v) Changing play with a sword to play with a plane (vi) Replacement dog feeding activity with bird feeding

## Data Availability

The data used to support the findings of this study is available only to the authors, in order to protect participants' privacy.
